The article "Identification of Key Genes Related to the Obesity Patients with Osteoarthritis Based on Weighted Gene Coexpression Network Analysis (WGCNA)" was retracted in 2023. Reasons: signs of a paper mill; compromised peer review; unreliable results or conclusions.

# Identification of Key Genes Related to the Obesity Patients with Osteoarthritis Based on Weighted Gene Coexpression Network Analysis (WGCNA)

**DOI:** 10.1155/2022/8953807

**Published:** 2022-07-11

**Authors:** Quan Zhou, Huan Sun, Jin Jia, Jun-liang Jiang, Tao Li, Zhao-xiang Wu, Zhong Chen

**Affiliations:** ^1^Department of Orthopedics, The First People's Hospital of Dali City, Dali, Yunnan 671000, China; ^2^Department of the Basic Medicine, The Kunming Medical University, Kunming, Yunnan 650500, China; ^3^Department of Orthopedics and Trauma, The Affiliated Hospital of Yunnan University (The Second People's Hospital of Yunnan Province, The Eye Hospital of Yunnan Province), Kunming, Yunnan 650000, China

## Abstract

**Background:**

Increasing evidence has suggested that obesity affects the occurrence and progression of osteoarthritis (OA). However, the underlying molecular mechanism that obesity affects the course of OA is not fully understood and remains to be studied.

**Methods:**

The gene expression profiles of the GSE117999 and GSE98460 datasets were derived from the Gene Expression Omnibus (GEO) database. Firstly, we explored the correlation between obesity and OA using chi-square test. Next, weighted gene coexpression network analysis (WGCNA) was executed to identify obesity patients with OA- (obesity OA-) related genes in the GSE117999 dataset by “WGCNA” package. Moreover, differential expression analysis was performed to select the hub genes by “limma” package. Furthermore, ingenuity pathway analysis (IPA) and functional enrichment analysis (“clusterProfiler” package) were conducted to investigate the functions of genes. Finally, the regulatory networks of hub genes and protein-protein interaction (PPI) network were created by the Cytoscape 3.5.1 software and STRING.

**Results:**

A total of 15 differentially expressed obesity OA-related genes, including 9 lncRNAs and 6 protein coding genes, were detected by overlapping 66 differentially expressed genes (DEGs) between normal BMI samples and obesity OA samples and 451 obesity OA-related genes. Moreover, CCR10, LENG8, QRFPR, UHRF1BP1, and HLA-DRB4 were identified as hub genes. IPA results indicated that the hub genes were noticeably enriched in antimicrobial response, inflammatory response, and humoral immune response. PPI network showed that CCR10 interacted more with other proteins. Gene set enrichment analysis (GSEA) indicated that the hub genes were related to protein translation, cancer, chromatin modification, antigen processing, and presentation.

**Conclusion:**

Our results further demonstrated the role of obesity in OA and might provide new targets for the treatment of obesity OA.

## 1. Background

Osteoarthritis (OA) is a systemic joint disease characterized by joint dysfunction as well as chronic disability. The pathological manifestation is the degeneration of the inner weight-bearing compartment of cartilage, which involves the structural changes of hyaline articular cartilage, subchondral bone, ligament, joint capsule, synovium, and surrounding muscles. Cartilage degeneration is the end-stage sign of the disease [1]. The incidence of knee OA is 10%-60% in the United States, and about 13% of them are women [2]. Although the clinical treatment of OA contains drugs, physical therapy, and exercise therapy, they have not achieved very good therapeutic results. Therefore, it is especially necessary to develop new therapeutic targets for OA.

Obesity refers to the excessive accumulation of fat in the body, resulting in a disease that exceeds the normal weight, which is closely related to a variety of diseases [3]. Obesity and OA are two common health problems in the world. The latest research has indicated that obesity affects the occurrence and development of OA [4–7]. Moreover, it has been revealed that obesity is a risk element for OA, especially in weight-bearing joints [8]. However, this relationship does not explain OA in nonweight bearing joints, for instance, hand OA and shoulder OA. Furthermore, metabolic inflammation caused by obesity has been regarded as a key factor in the pathogenesis of OA [9]. On the other hand, obesity can also affect the regulation of glucose tolerance and fat metabolism pathway, resulting in osteosclerosis, cartilage matrix rupture, or OA [10]. In addition, adipose tissue can also affect the process of OA because it can be the main source of metabolic active medium of cytokines, chemokines, and adipokines [11]. Adipokines such as adiponectin and leptin have been suggested to be involved in the regulation of inflammatory and immune response of cartilage. Inflammatory cytokines released by adipose tissue can negatively regulate cartilage, eventually inhibiting the synthesis of proteoglycan and type II collagen by activating the production of other cytokines and matrix metalloproteinases along with prostaglandins [12]. Therefore, inflammatory cytokines released by adipose tissue take a key role in cartilage matrix degradation and bone resorption of OA. However, the underlying molecular mechanism of obesity patients with OA (obesity OA) is not entirely clear.

For this study, we intended to explore the molecular mechanisms of obesity OA by comprehensively bioinformatic analyses. Firstly, we compared the relationship between BMI value and OA. Next, weighted gene coexpression network analysis (WGCNA) was performed to screen obesity OA-related genes. Moreover, ingenuity pathway analysis (IPA) and functional enrichment analysis were performed to investigate the functions of genes. Therefore, this study may provide reference for the prevention and treatment of obesity OA.

## 2. Materials and Methods

### 2.1. Data Acquisition

OA-related datasets (GSE117999 and GSE98460) were downloaded from the Gene Expression Omnibus (GEO) database (http://www.ncbi.nlm.nih.gov/geo), which includes transcriptional data and clinical information. The GSE117999 dataset includes 12 knee cartilage samples of OA patients and 12 knee cartilage samples of patients with arthroscopic partial meniscectomy (control samples), while the GSE98460 dataset contains 20 tibial plateau cartilage samples of obesity OA and 3 tibial plateau cartilage of nonobesity OA.

### 2.2. Relationship of Obesity and OA

To explore the relationship of obesity and OA, we compared the differences of age, sex, and BMI between OA and non-OA patients by combining the data from the GSE117999 and GSE98460 datasets using the chi-square test.

### 2.3. Gene Set Enrichment Analysis (GSEA)

To recognize the differential signaling pathway associated with obesity OA, GSEA was performed in the GSE117999 dataset using the “clusterProfiler” R package [13]. *p* < 0.05 and false discovery rate (FDR) < 0.05 were regarded as statistically significant.

### 2.4. Weighted Gene Coexpression Network Analysis (WGCNA)

WGCNA was undertaken by “WGCNA” package in R [14]. Firstly, we selected the samples, including normal and OA samples, with the value of BMI greater than 27 as obesity patients from the GSE117999 dataset. Next, gene expression matrix of obesity samples was extracted for WGCNA. Subsequently, sample clustering analysis was performed to remove the outlier samples by using the hclust function. Moreover, expression correlation between any two genes was analyzed by Pearson correlation analysis, and the weighting coefficient was at least 0.8. Furthermore, we transformed the matrix of expression correlation into an adjacency matrix, and the adjacency matrix was transformed into the topological overlap matrix (TOM) which was used to assess the interconnection between any two genes. Finally, the corresponding dissimilarity (1-TOM) was calculated to confirm hierarchical clustering nodes with modules, and modules with similar expression pattern were segmented by dynamic tree cutting algorithm.

The module with the highest absolute value of correlation coefficient between the module eigengene (ME) and the clinical traits and *p* < 0.05 was defined as key module. In addition, the key genes with the absolute value of correlation coefficient more than 0.6 in the key module were selected and defined as obesity OA-related genes for subsequent analysis.

### 2.5. Identification of Differentially Expressed Genes (DEGs)

The “limma” package was utilized to identify DEGs between normal BMI samples and obesity OA from the GSE117999 dataset, and the threshold criterion was set as ∣log FC | >1 and *p* value < 0.05 [15]. Then, heat map and volcano plot of DEGs were drawn by the “pheatmap” package and ggplot package [16]. In addition, Venn diagram was adopted to screen the differentially expressed obesity OA-related genes by overlapping the DEGs and obesity OA-related genes.

### 2.6. Validation of the Expression of the Differentially Expressed Obesity OA-Related Genes

To verify the expression levels of the differentially expressed obesity OA-related genes, log-rank tests and box plots were used to compare the expression levels of these protein coding genes between normal and obesity OA samples and between obesity non-OA and obesity OA samples in the GSE117999 dataset. Moreover, we also compared the significant differences between normal BMI samples and obesity OA in the GSE98460 dataset and visualize the differences, respectively. Moreover, the differentially expressed obesity OA-related genes in GSE98460 dataset with statistical difference were defined as the hub genes for subsequent analysis.

### 2.7. Ingenuity Pathway Analysis (IPA) and Protein-Protein Interaction (PPI) Network

For exploring the disease and function pathways of DEGs, the ingenuity pathway analysis (IPA) was performed. In addition, the heat map was further used to visualize the activated or inhibited pathways using the expression matrix of the hub genes. Moreover, to search for the regulated pathway of DEGs, the upstream and downstream regulatory networks of the hub genes were constructed by the Cytoscape 3.5.1 software. On the second hand, a PPI network of hub genes and other proteins was further constructed to verify their interaction relationship with the help of STRING (https://string-db.org/) and Cytoscape 3.5.1 [17].

### 2.8. Functional Enrichment Analysis

In order to explore biological processes and signaling pathways related to the hub genes, GSEA was performed through the “clusterProfiler” package based on the expressed data of GSE98460 [13]. A *p* value < 0.05 was considered as a statistically significant enrichment.

## 3. Results

### 3.1. Relationship of Obesity and OA

To confirm the relationship between obesity and OA, we compared the levels of age, sex, and BMI in OA and non-OA patients by chi-square test. As seen in Table 1, patients with higher obesity morbidity and older age were discovered in the OA patients compared than control group, suggesting that obese people may be more prone to OA.

### 3.2. GSEA Analysis

In order to explore biological processes and signaling pathways associated with the obesity OA. GSEA was performed in the GSE117999 dataset. As expected, genes in the obesity OA were primarily linked to the metabolism-related pathways, such as glycerolipid metabolism, starch and sucrose metabolism, nicotinate and nicotinamide metabolism, and retinol metabolism (Figure 1), indicating that metabolic imbalance possible essential role in obesity OA.

### 3.3. WGCNA

For screening the significant genes related to obesity OA, WGCNA was utilized to identify the genes with highly similar expression forms in the modules; the optimum soft threshold was selected as 19 (Figure 2(a)). Then, by setting MEDissThres as 0.2, a sum of 23 modules were confirmed by dynamic tree cutting algorithm (Figure 2(b)). Furthermore, correction analysis suggested that the MEplum4 module was defined as the obesity OA-related module (Cor = 0.88 and *p* < 0.05, Figure 2(c)). Finally, 439 genes with the absolute value of correlation coefficient beyond 0.6 and *p* value < 0.5 were identified as obesity OA-related genes (Figure 2(d)).

### 3.4. Identification of the Differentially Expressed Obesity OA-Related Genes

A total of 66 DEGs (38 downregulated and 28 upregulated genes) were identified between normal BMI samples and obesity OA. The heat map and volcano plot of these DEGs are shown in Figures 3(a) and 3(b), respectively. In addition, 15 differentially expressed obesity OA-related genes were identified by overlapping 66 DEGs and 451 obesity OA-related genes (Figure 3(c)). Notably, among the 15 differentially expressed ORGs, 9 genes were lncRNAs, while the remaining 6 genes can code proteins. Thus, we selected these 6 genes for subsequent analysis.

### 3.5. Verification the Expression of Protein Coding Genes

To further confirm the expression levels of these 6 protein coding genes, we firstly compared the expression levels of these 6 protein coding genes between normal and obesity OA samples and between obesity non-OA and obesity OA samples in the GSE117999 dataset. The results indicated that 5 protein coding genes, including CCR10, HLA-DRB4, LENG8, QRFPR, and UHRF1BP1, were shown significant differences between obesity non-OA and obesity OA samples (Figure 4(a)), while the remaining genes had no statistic difference between these two groups. Interestingly, we found that CCR10, QRFPR, and UHRF1BP1 are upregulated in obesity OA samples compared to normal samples and in obesity OA samples compared to obesity non-OA samples, but LENG8 and HLA-DRB4 are downregulated (Figures 4(a) and 4(b)). However, the results of GSE98460 showed that CCR10, HLA-DRB4, LENG8, QRFPR, and UHRF1BP1 had no significance between obesity non-OA and obesity OA samples (Figure 4(c)), which might be due to the limited sample size because the GSE98460 dataset only includes 3 obesity non-OA samples and their BMI values were 27. Therefore, CCR10, HLA-DRB4, LENG8, QRFPR, and UHRF1BP1 were regarded as the hub genes.

### 3.6. IPA

To further explore the disease and functional pathways of DEGs, IPA was further conducted. The results revealed that DEGs were mostly associated with the antimicrobial response, inflammatory response, and humoral immune response pathways (Figure 5(a)). Moreover, as shown in Figure 5(b), inflammatory response, chemotaxis, cell death of leukemia cell lines, and lymphocyte migration pathways were activated, while the inflammation of organ, extracranial solid tumor, and recruitment of granulocyte pathways were inhibited. Furthermore, the upstream and downstream regulatory networks displayed that the hub genes were involved in the regulation of the enzyme, kinase, and ligand-dependent nuclear receptor (Figures 5(c) and 5(d)).

### 3.7. PPI Network

To explore the interaction between the proteins and the hub genes, the PPI network of these hub genes was constructed by using the STRING database. As shown in Figure 6, the CCR10 interact more with other proteins.

### 3.8. Functional Analysis

GSEA was chosen to discover the underlying molecular mechanisms of these 5 hub genes. As shown in Figures 7(a) and 7(b), GSEA suggested that CCR10 was mainly involved in biological processes of cotranslated protein targeting to membrane, protein localization to endoplasmic reticulum, and mainly related to ribosomes, colorectal cancer, and cancer pathways. Moreover, QRFPR was mainly enriched in covalent chromatin modification, detection of stimuli related to sensory perception, Golgi vesicular transport biological processes and olfactory conduction, and pyrimidine metabolism pathways (Figures 7(c) and 7(d)).

## 4. Discussion

Obesity is a dominant and independent risk indicator for OA [18, 19]. Obesity can contribute to both weight-bearing as well as non-weight-bearing OA. The weight load caused by obesity can bring excess load to the load-bearing joint, which may cause uneven stress on the joint surface and joint dysfunction, further leading to cartilage loss, osteophyte formation, and OA [20]. From a nonweight bearing viewpoint, hand joint OA is caused by metabolic changes, such as abnormal lipid metabolism, abnormal glucose tolerance, and hyperuricemia, which are resulted by obesity [21]. In addition, OA can cause obesity. For example, the pain caused by OA will limit and reduce physical activity, thus further increasing the risk of weight, inflammation, and cardiovascular disease [19]. However, the common molecular mechanism of obesity OA is still not well understood.

In this study, we analyzed the GSE117999 dataset from the GEO database and found that CCR10, HLA-DRB4, LENG8, QRFPR, and UHRF1BP1 may play key roles in obesity OA; however, we did not achieve the same results in GSE98460 database because of the limited sample size. LENG8 (Leukocyte Receptor Cluster Member 8) is a protein-coding gene that is essential in the immune response [22], renal carcinoma, and blood brain barrier and brain signal transduction [23, 24]. HLA-DRB4 is mainly used for immune antigen matching in organ and bone marrow transplantation [25] and also is instrumental in the development of type 1 diabetes (T1D), cellular disease (CD) [26], periodontitis [27], and rheumatoid arthritis [28]. In addition, recent studies suggested that HLA-DRB4 is also a hereditary risk driver for Churg-Strauss syndrome (CSS), resulting in increasing the possibility of CSS vasculitis [29]. In addition, HLA-DRB4 was localized in the neighboring 6p21 region [30], and the genes localized in this part of the genome showed high expression in the adipose tissue [31]. UHF1BP1 is a risk factor for systemic lupus erythematosus and has a major function in a variety of tumors [32–34]. Moreover, UHF1BP1 is also involved in the development of neurodevelopmental disorders leading to the obsessive-compulsive disorder (OCD) [35].

CCR10 is a member of the chemokine receptor subfamily and is originally secreted in blood leukocytes as a fraction of CD4 and CD8 memory T cells [36]. It has been revealed that CCR10 is overexpressed in a variety of tumors [37]. CCR10 has been suggested to be related to skin immune diseases [38], respiratory allergic diseases [39], angiogenesis, and wound healing [40]. In addition, human CCR10 promoter is coactivated by Ets-1 and vitamin D receptor in the presence of 1,25-(OH) 2D3, and vitamin D metabolism in vivo is closely related to bone production and repair [41]. The RFamide neuropeptide family of pyroglutamylated RFamide peptide (QRFP) is engaged in a wide-range of biological activities, and it can bind to its receptor GPR103 and influences various biological functions which extending from food intake and cardiovascular functioning to analgesia, aldosterone secretion, neurodevelopment, eclampsia, locomotor activity, and reproduction [42–44]. The latest research showed QRFP regulates glucose homeostasis and bone mineralizationl [45]. Especially in Osteogenesis imperfecta (OI), QRFPR plays a remarkably significant function in its occurrence and development [46]. Therefore, it is possible that these genes could serve a critical function in obesity OA.

Moreover, the results of PPI network showed that CCR10 and QRFPR proteins interacted more closely with other proteins. Combined with IPA analysis, we found that they were related to many disease pathways, which suggested that they could play more roles in obesity OA. In addition, we further analyzed the pathways involved in CCR10, HLA-DRB4, LENG8, QRFPR, and UHRF1BP1 through GSEA. Among them, CCR10 was mainly enriched in the biological processes of cotranslated protein targeting to membrane and protein localization to endoplasmic reticulum. KEGG results suggested that CCR10 was mainly associated with ribosomes, colorectal cancer, and cancer pathways. QRFPR was mainly enriched in covalent chromatin modification, detection of stimuli related to sensory perception, Golgi vesicular transport biological processes and olfactory conduction, and pyrimidine metabolism pathways. These results suggested that CCR10 and QRFPR may play a central effect in obesity OA by regulating these biological processes and pathways. Though we have screened five potential candidate obesity OA-related genes using bioinformatics technology, our study still has limitations. First, we did not include other health conditions to differentiate hub genes because lack of the clinical follow-up information in the samples. Second, the results achieved by bioinformatics analysis only were insufficient, which need to be confirmed by experimental verification. Therefore, it is necessary to carry out further genetic and experimental research on larger samples and carry out experimental verification.

## 5. Conclusions

In this study, we identified CCR10, HLA-DRB4, LENG8, QRFPR, and UHRF1BP1 as the hub genes in obesity OA based on the GSE117999 and GSE98460 datasets. Moreover, we also further investigated the function of CCR10, HLA-DRB4, LENG8, QRFPR, and UHRF1BP1. Thus, CCR10, HLA-DRB4, LENG8, QRFPR, and UHRF1BP1 may act as biomarkers of obesity OA. Therefore, these findings may be helpful in increasing the knowledge of the molecular mechanisms responsible for obesity. However, the mechanisms underlying the roles of CCR10, HLA-DRB4, LENG8, QRFPR, and UHRF1BP1 in obesity OA remain unknown. Thus, additional research is needed to elucidate these mechanisms.

## Figures and Tables

**Figure 1:** The GSEA results obtained by GSEA 4.0.3 in the GSE117999 dataset.

**Figure 2:** Identification of obesity OA-related genes based on WGCNA in the GSE117999 dataset. (a) Determination of the optimal soft threshold to conform to the scale-free distribution. (b) Dendrogram of genes clustered based on the highly correlated eigengenes. (c) Correlations between modules and obesity OA. (d) 439 genes with the correlation coefficient over 0.6 and *p* value < 0.5 were identified as obesity OA-related genes.

**Figure 3:** Recognition of the differentially expressed obesity OA-related genes in the GSE117999 dataset. (a) The heat map of DEGs between normal BMI samples and obesity OA. (b) The volcano plot of DEGs between normal BMI samples and obesity OA. (c) 15 differentially expressed obesity OA-related genes were screened by overlapping 66 DEGs and 451 OA-related genes.

**Figure 4:** The expression of CCR10, HLA-DRB4, LENG8, QRFPR, and UHRF1BP1 between obesity non-OA and obesity OA samples (a), between normal and obesity OA samples (b) in the GSE117999 dataset, and between obesity non-OA and obesity OA samples (c) in the GSE98460 dataset.

**Figure 5:** The IPA results obtained by IPA 01-19-02 in the GSE117999 dataset. (a) DEGs were mainly associated with the antimicrobial response, inflammatory response, and humoral immune response pathways. (b) Inflammatory response, chemotaxis, cell death of leukemia cell lines, and lymphocyte migration pathways were activated, while the inflammation of organ, extracranial solid tumor, and recruitment of granulocyte pathways were inhibited. (c, d) The upstream and downstream regulatory networks displayed that the hub genes were involved in the regulation of the enzyme (c), kinase, and ligand-dependent nuclear receptor (d).

**Figure 6:** The PPI network of hub genes obtained by Cytoscape 3.5.1.

**Figure 7:** The functional enrichment analysis of CCR10 and QRFPR. (a) CCR10 was mainly involved in biological processes of cotranslated protein targeting to membrane and protein localization to endoplasmic reticulum. (b) CCR10 was mainly related to ribosomes, colorectal cancer, and cancer pathways. (c) QRFPR was mainly enriched in biological processes of covalent chromatin modification, detection of stimuli related to sensory perception, and Golgi vesicular transport. (d) CCR10 was mainly related to olfactory conduction and pyrimidine metabolism pathways.

**Table 1:** Comparison of the levels of age, sex, and BMI in OA and non-OA patients.

	Age (years)		Gender		Obesity	
	≥ 60	<60	Female	Male	BMI > 27	BMI ≤ 27
OA	39	39	35	23	52	6
Non-OA	2	9	5	7	6	6
*p* value	0.009		0.3845		0.003767	

## Data Availability

All data, models, and code generated or used during the study appear in the submitted article.
